The article "The longitudinal relationship between tourism, electricity consumption, and CO2 emissions" was retracted in 2025. Reasons: unreliable results or conclusions; concerns about the authorship.

# The longitudinal relationship between tourism, electricity consumption, and CO_2_ emissions

**DOI:** 10.1016/j.heliyon.2024.e35724

**Published:** 2024-08-20

**Authors:** Rizwan Munir, Tahir Abbas, Liaqat Ali Waseem, Jiliang Sheng, Wang Jing, Mohammad Abid, Muneeb Ahmad, Mohammad K. Okla

**Affiliations:** a School of Statistics and Data Science, Jiangxi University of Finance and Economics, Nanchang, China; b Department of Mathematics, College of Sciences, University of Sharjah, Sharjah, 0000, United Arab Emirates; c Department of Geography, Government College University Faisalabad, Pakistan; d Department of Statistics, Government College University, Faisalabad, Pakistan; e Botany and Microbiology Department, College of Science, King Saud University, P.O. Box 2455, Riyadh, 11451, Saudi Arabia

**Keywords:** Tourism industry, electricity use, Intercountryal trade, Foreign direct investment, ARDL, FMOLS, DOLS, Pakistan

## Abstract

The objective of the study is to determine the electricity use, and tourism industry environmental impacts, and increase in CO_2_ emissions in Pakistan. What are the linkages of foreign direct investment, intercountryal trade, gross domestict product, and CO_2_ emissions. The study has applied the Autoregressive distributed lag (ARDL) method to analysis the data set from 1985 to 2023. The robustness test is applied using Dynamic Ordinary Least Square (DOLS), and Fully modified ordinary least squares (FMOLS). The results reveal that the increase in the electricity use, and tourism industry has significant negative impacts on CO_2_ emissions in both short- and long-run. The increase in intercountry trade effects the Domestic Product growth (GDP) growth and causes to increase in use of fossil fuels, which are the major source of CO_2_ emissions. The increase in foreign direct investment (FDI) increase the GDP growth, and FDI also increase the CO_2_ emissions in Pakistan. The results suggests that the incresae in the renewal energy consumption for the electricity production and transportation can help to decrease the CO_2_ emissions in Pakistan.

## 1 Introduction

Greenhouse gas emissions, especially CO_2_, threaten the environment's long-run sustainability, development, and health. Pakistan is a tourism hub with a strong economy and growing agriculture. Considering the summit's objective of achieving a 50 % reduction in greenhouse gas emissions by 2050, it is imperative for the travel and tourist sector to transition towards a low-carbon economy and significantly decrease its CO_2_ emissions [1]. The travel industry is one of the most vocal advocates for a low-carbon economy [2]. Environmental pollution is positively and significantly impacted by both GDP and electricity usage [3]. There is a clear relationship between the use of ICT, electricity consumption, CO_2_ emissions, and GDP growth [4]. There is a notable correlation between trade policy variables and exports and imports [5]. The globalisation, energy usage, trade, and GDP growth have positive connections with the ecological footprint [6]. There is a strong correlation between FDI inflow and CO_2_ emissions in the long run [7]. There is a correlation between economic growth and environmental pollution, specifically in terms of regional GDP growth and the sustainability of SO_2_ emissions [8]. The objectives of the study are to investigate the relationships between the tourism industry, electricity use, GDP growth, FDI, and CO_2_ emissions in Pakistan. The research also evaluates the relationship between tourism industry, and energy use in both short- and long-run. The study has applied the DOLS, FMOLS, and ARDL models to analyze the data and found the answers of the following research questions: a) What is the impact of electricty production increase on CO_2_ emissioms. b) How GDP growth create changes in environmental pollution rate. What are the impacts of FDI, and tourism industry on environmental pollution in Pakistan. The results reveal that the tourism industry and electricity use have significantly negative impacts on CO_2_ emissions in long-run. FDI investment has significant positive impact onenvironmental changes in Pakistan. In order to propose policy enlightenment grounded in diversity.

The article "The longitudinal relationship between tourism, electricity consumption, and CO2 emissions" was retracted in 2025. Reasons: unreliable results or conclusions; concerns about the authorship.

The paper's succeeding parts follow this structure: Section 2 reviews all relevant scholarly literature about the topic. section 3 describes the study's data collection and econometric methods. Section 4 presents and analyses study findings. Section 5 concludes the study results and provides future research suggestions.

## 2 Literature review

According to Ref. [9], while tourism and economic development raise CO_2_ emissions in Turkey, the use of renewable energy sources and increased agricultural production lower CO_2_ emissions. The sustainable growth in tourism industry has significant positive on economies of China and France [10]. [11] found a U-shaped relationship between tourism industry growth, and PM_2.5_ emissions in central and western China. The most significant factors influencing air pollution are GDP and industrial structure [12]. [13] found that the transportation use for tourism industry increased the CO_2_ emissions. The environmental Kuznets curve (EKC) illustrated an inverted U-shaped relationship between tourism industry and air pollution [14]. According to Ref. [15], there is a negative association between tourism and CO_2_ emissions, and the tourist sector has significantly worsened environmental pollution in 27 European nations. As per [16], the expansion of the tourist sector leads to a corresponding rise in CO_2_ emissions [17]. the higher tourism densities were associated with reduced greenhouse gas emissions and better environmental performances. The electricity production using fossil fuels has significant negative impacts on environmental pollution in China [18]. A study discovered a link between electricity production, industrial energy usage, and environmental pollution in the industrial efficiency of different provinces in China. There exists a direct relationship between long-term electricity consumption and CO_2_ emissions [19]. It has been observed that there is a direct correlation between the use of renewable energy and CO_2_ emissions [20]. A study discovered a significant link between electricity usage, economic development, and environmental pollution across 35 OECD countries [21]. Based on research, public-private partnership investments in energy consumption have been found to have negative impacts on CO_2_ emissions in India [22]. Most of the electricity in Kuwait is generated from fossil fuel sources to meet industrial demands, resulting in a significant rise in CO_2_ emissions [23]. The increase in CO_2_ emissions was caused by the energy consumption in electricity production [24]. A study discovered a correlation between electricity consumption and CO_2_ emissions in Brazil, indicating a negative relationship [25]. A study discovered a significant correlation between the growth of GDP and the sustainability of SO_2_ emissions [26]. The relationship between GDP, energy consumption intensity, and SO_2_ emissions was found to be unidirectional, with each factor influencing the others [27]. A study discovered a U-shaped correlation between economic growth and environmental changes [28]. The rise in economic growth leads to a surge in fossil fuel consumption, resulting in a corresponding increase in CO_2_ emissions [29]. [30] applied the ARDL model and discovered a favourable connection between economic growth, energy usage, urbanisation, and CO_2_ emissions in MINT countries. As stated in Ref. [31], the growth of the economy and the development of the tourism industry have a notable adverse effect on CO_2_ emissions. A study discovered that economic growth had a notable adverse effect on environmental pollution [32]. The economic development has led to a significant increase in environmental pollution, both in the short and long term [33]. The GDP growth had a noticeable adverse effect on environmental pollution [34]. The FDI inflows contributed to the economic growth, resulting in a notable reduction in CO_2_ emissions [35]. The impacts of tourism, urbanisation, and financial expansion on CO_2_ emissions are all impacted by FDI [36]. Both FDI inflows and GDP growth were positively impacted by FDI inflows, which also raised CO_2_ emissions [37]. There is a one-way causal relationship between FDI and carbon emissions, and [38] indicates that FDI significantly reduced CO_2_ emissions. India's CO_2_ emissions have decreased as a consequence of the growth in FDI inflows and the usage of renewable energy [39]. discovered a favourable correlation between FDI and renewal energy [40]. Additionally, it found that using more renewable energy reduced CO_2_ emissions. There was a negative correlation, per [41], between FDI and contamination of the environment. FDI inflow and environmental pollution were shown to be negatively correlated by Ref. [42] after using the two-step system GMM model. A unidirectional association between the intercountry tourist business, energy consumption, and CO_2_ emissions was verified by the Granger causality test [43]. Intercountry commerce leads to higher GDP per capita, which in turn causes higher CO_2_ emissions [44]. There is a strong inverse link between international trade and environmental contamination, according to Ref. [45]. On the other hand [46], discovered that the rise in commerce significantly reduced CO_2_ emissions. Increased industrial expansion is a result of increased international trade and FDI inflows, which raises CO_2_ emissions [47]. [48] discovered that China's CO_2_ emissions rose together with the growth in international commerce. Short- and long-term reductions in environmental contamination are brought about by the expansion of international commerce [49]. Environmental contamination rises with increased international commerce [50]. Compared to OECD nations, APEC countries have greater environmental degradation consequences from international commerce [51].

The article "The longitudinal relationship between tourism, electricity consumption, and CO2 emissions" was retracted in 2025. Reasons: unreliable results or conclusions; concerns about the authorship.

## 3 Methods and techniques

### 3.1 Data collection

The present investigation employed yearly data pertaining to the dependent variable, CO_2_ emissions, as well as the independent variables, namely electricity consumption (EC), Gross GDP, FDI, intercountryal trade (IT), and tourism industry (TOUR), spanning the years 1985–2022. Quantifying environmental harm encompasses the monitoring of CO_2_ emissions, whilst measuring economic progress entails the examicountry of GDP growth. CO_2_ emissions refer to the quantity of carbon dioxide released into the atmosphere as a result of human activities, primarily the combustion of fossil fuels. The variable that is influenced by other factors in this particular situation is carbon dioxide emissions, which are discharged into the atmosphere as a result of the combustion of fossil fuels. Table 1 displays the symbols used to represent variables and the sources of the data.

**Table 1:** Denotes the specific information and sources used for collecting data.

Variables deatil	Symbols	Sources
Foreign direct investment	FDI	https://data.worldbank.org.com
Gross domestic product (USD $)	GDP	https://data.worldbank.org.com
Intercountryal trade volume of the country	IT	https://data.worldbank.org.com
Energy used (in shape of Oil and Coal) for electricity production	EC	https://data.worldbank.org.com
Carbon dioxide emissions in tonnes	CO_2_	https://data.worldbank.org.com
Tourism industry	TOUR	https://data.worldbank.org.com

Several key factors drive the selection of CO_2_ emissions as the dependent variable and the chosen independent variables, which include EC, GDP, FDI, IT, and TOUR. To begin with, CO_2_ emissions serve as a vital measure of the environmental consequences, specifically in relation to global warming and climate change. Furthermore, these factors have a strong correlation with economic development, rendering them vital for comprehending the environmental ramifications of economic development.

### 3.2 Econometrical farmework

Here is the fundamental econometric model that was utilised for the research:

(1) $${\text{CO}}_{2}=f\;\left(\text{EC},\text{TOUR},\text{FDI},\text{GDP},\text{IT}\right)$$

All variables have their stationarity changed using logarithms (ln). Log-quadratic regression is used to get Equation (1):

(2) $${\text{lnICO}}_{2t}=\alpha_{0}+\beta_{1}\;\text{lnFDI}+\beta_{2}\;\text{lnEC}+\beta_{3}\;\text{lnTOUR}+\beta_{4}\;\text{lnGDP}+\beta_{5}\;\text{lnIT}+є$$

Equation (2) predicted signs include positive values for β_1_, β_2_, β_3_, and β_4_. Since the EKC model takes tourism and FDI into account, the number of tourisms has a direct influence on CO2 emissions. The ARDL cointegration approach does not necessitate a panel unit root pre-assessment as it allows for testing cointegration among a set of variables with different orders of integration as I (0) and I (1). Where "ε_t_" is the error run, β′s are the slope parameters. CO_2t_, lnFDI, lnEC, lnTOUR, lnGDP, lnIT, are the natural Log of no variables must be included in I (2) because this would invalidate the procedure.

### 3.3 Cointegration test

Limits analysis and Johansen cointegration are used to examine the variables' long-term connection. While Equation (2) is constructed to do cointegration using the ARDL technique, and Equation (3) is as follows,:

(3) $${\text{lnCO}}_{2t}=\alpha_{0}+\sum_{i=1}^{p_{1}}\beta_{i}\Delta \ln\;{\text{CO}}_{2t-i}+\sum_{i=0}^{p_{2}}\gamma_{i}{\Delta \text{lnFDI}}_{t-i}+\sum_{i=0}^{p_{3}}\rho_{i}{\Delta \text{lnGDP}}_{t-i}+\sum_{i=0}^{p_{4}}\vartheta_{i}{\Delta \text{lnIT}}_{t-i}^{2}+\sum_{i=0}^{p_{5}}\mu_{i}{\Delta \text{lnFDI}}_{t-i}+\sum_{i=0}^{p_{6}}\pi_{i}{\Delta \text{lnTOUR}}_{t-i}+\Phi_{11}{\text{lnCO}}_{2t-1}+\Phi_{12}{\text{lnEC}}_{t-1}+\Phi_{13}{\text{lnGDP}}_{t-1}+\theta_{14}\;\ln\;{\text{IT}}_{t-1}+\Phi_{15}{\text{lnFDI}}_{t-1}+\Phi_{16}{\text{lnTOUR}}_{t-1}+\varepsilon_{t}$$

Where β_i_, γ_i_, ρ_i_, θ_i_, λ_i_, π_i_, Φ_11_, Φ_12_, Φ_13_, Φ_14_, Φ_15_, and Φ_16_ are the estimated parameters, and Δ signifies the 1st difference between the variables. Akaike's information criterion (AIC) derunines the appropriate lag lengths of p_1_, p_2_, p_3_, p_4_, and p_5_, where ε_t_ represents the error terrm. F-statistics are used in the primary phase of the ARDL model's error correction procedure to analyze the variables. Both presumptions acknowledge that I (0) and I (1) are the only autoregressive distributed slack approach variables. Equation (4) for the F-statistic test states the null and alternative hypotheses in the following manner:

$$H_{0}:\left(\varphi_{1}=\varphi_{2}=\ldots =\varphi_{k}=0\right);\;H_{1}:\left(\varphi_{1}=0,=\varphi_{2}=0\right)$$

(4) $${\Delta \text{lnCO}}_{2t}=\alpha_{0}+\sum_{i=1}^{p_{1}}\beta_{i}\Delta \ln\;{\text{CO}}_{2t-i}+\sum_{i=0}^{p_{2}}\gamma_{i}{\Delta \text{lnEC}}_{t-i}+\sum_{i=0}^{p_{3}}\delta_{i}{\Delta \text{lnGDP}}_{t-i}+\sum_{i=0}^{p_{4}}\vartheta_{i}{\Delta \text{lnGDP}}_{t-i}^{2}+\sum_{i=0}^{p_{5}}\mu_{i}{\Delta \text{lnFDI}}_{t-i}+\sum_{i=0}^{p_{6}}\pi_{i}{\Delta \text{lnTA}}_{t-i}+ℶ\;\text{ECT}+\varepsilon_{t}$$

The second-stage estimations and the long-run coefficient are determined. The estimation of the long-run coefficients is modified. The coefficient of the error term of the dependent variable is influenced by the corrective limitation on the extended equilibrium measure [52].

The article "The longitudinal relationship between tourism, electricity consumption, and CO2 emissions" was retracted in 2025. Reasons: unreliable results or conclusions; concerns about the authorship.

### 3.4 Granger causality

To evaluate causatives, the study uses cointegration and Granger causation with error correction [53]. Equation (6) will lead to a bigger Granger causality evaluation with error correction, the following equation (6) will be as follows:

(5) $$\left(\begin{array}{c} \begin{array}{c} {\text{lnCO}}_{2t}\\ {\text{lnGDP}}_{t} \end{array}\\ \ln\;{\text{IT}}_{t}\\ {\text{lnEC}}_{t}\\ {\text{lnFDI}}_{t}\\ {\text{lnTOUR}}_{t} \end{array}\right)=\left(\begin{array}{c} \lambda_{1}\\ \lambda_{2}\\ \lambda_{3}\\ \lambda_{4}\\ \lambda_{5}\\ \lambda_{6} \end{array}\right)+\left(\begin{array}{c} \sigma_{11,1}\;\sigma_{12,1}\;\sigma_{13,1}\;\sigma_{14,1}\;\sigma_{15,1}\;\sigma_{16,1}\\ \sigma_{21,1}\;\sigma_{22,1}\;\sigma_{23,1}\;\sigma_{24,1}\;\sigma_{25,1}\;\sigma_{26,1}\\ \sigma_{31,1}\;\sigma_{32,1}\;\sigma_{33,1}\;\sigma_{34,1}\;\sigma_{35,1}\;\sigma_{36,1}\\ \sigma_{41,1}\;\sigma_{42,1}\;\sigma_{43,1}\;\sigma_{44,1}\;\sigma_{45,1}\;\sigma_{46,1}\\ \sigma_{51,1}\;\sigma_{52,1}\;\sigma_{53,1}\;\sigma_{54,1}\;\sigma_{55,1}\;\sigma_{56,1}\\ \sigma_{61,1}\;\sigma_{62,1}\;\sigma_{63,1}\;\sigma_{64,1}\;\sigma_{65,1}\;\sigma_{66,1} \end{array}\right)\left(\begin{array}{c} \begin{array}{c} {\text{lnCO}}_{2t}\\ {\text{lnGDP}}_{t} \end{array}\\ \ln\;{\text{IT}}_{t}\\ {\text{lnEC}}_{t}\\ {\text{lnFDI}}_{t}\\ {\text{lnTOUR}}_{t} \end{array}\right)+\ldots +\left(\begin{array}{c} \sigma_{11,1}\;\sigma_{12,1}\;\sigma_{13,1}\;\sigma_{14,1}\;\sigma_{15,1}\;\sigma_{16,1}\\ \sigma_{21,1}\;\sigma_{22,1}\;\sigma_{23,1}\;\sigma_{24,1}\;\sigma_{25,1}\;\sigma_{26,1}\\ \sigma_{31,1}\;\sigma_{32,1}\;\sigma_{33,1}\;\sigma_{34,1}\;\sigma_{35,1}\;\sigma_{36,1}\\ \sigma_{41,1}\;\sigma_{42,1}\;\sigma_{43,1}\;\sigma_{44,1}\;\sigma_{45,1}\;\sigma_{46,1}\\ \sigma_{51,1}\;\sigma_{52,1}\;\sigma_{53,1}\;\sigma_{54,1}\;\sigma_{55,1}\;\sigma_{56,1}\\ \sigma_{61,1}\;\sigma_{62,1}\;\sigma_{63,1}\;\sigma_{64,1}\;\sigma_{65,1}\;\sigma_{66,1} \end{array}\right)\;\left(\begin{array}{c} \begin{array}{c} {\text{lnCO}}_{2t}\\ {\text{lnGDP}}_{t} \end{array}\\ \ln\;{\text{IT}}_{t}\\ {\text{lnEC}}_{t}\\ {\text{lnFDI}}_{t}\\ {\text{lnTOUR}}_{t} \end{array}\right)+\left(\begin{array}{c} \Phi_{1}\\ \Phi_{2}\\ \Phi_{3}\\ \Phi_{4}\\ \Phi_{5}\\ \Phi_{6} \end{array}\right)\;{\text{ECT}}_{t-1}+\left(\begin{array}{c} \varepsilon_{1,t}\\ \varepsilon_{2,t}\\ \varepsilon_{3,t}\\ \varepsilon_{4,t}\\ \varepsilon_{5,t}\\ \varepsilon_{6,t} \end{array}\right)$$

The ECT_t-1_ represents the examination of causality for both long- and short-term effects be statistically significant to environmental pollution, and ε_1_,_t_ to ε_6_,_t_ represents the stochastic standard errors.

### 3.5 Environmental kuznet curve

The updated Environmental Kuznets Curve (EKC) emerged from the necessity to incorporate ecological harm into the concept. Fig. 1 visually depicts the EKC, and Kuznets Bend shows how inequality and per capita income form a U-shaped.

**Fig. 1:** Graphical representation of the environmental Kuznets curve (EKC).

The additional of the reimbursement scattering pivot in the environmental Kuznets curve by expected environmental changes.

### 3.6 ARDL Model's diagnostic tests

Assuming normal distribution and serial independence for errors in Equation (3) is the fundamental idea behind the ARDL limits analysis technique. The Breusch-Godfrey serial correlation LM test, Ramsey reset test, and “Breusch-Pagan-Godfrey” test will be employed to assess heteroscedasticity and evaluate the model's working formula [54].

The article "The longitudinal relationship between tourism, electricity consumption, and CO2 emissions" was retracted in 2025. Reasons: unreliable results or conclusions; concerns about the authorship.

### 3.7 Robustness test

The study has created a pattern model using OLS regression to assess health of data analysis. The research has used the coint johansen capability of Python's statsmodels module to construct DOLS and FMOLS models for evaluating long-run coefficients. It splits the dataset into smaller subsets and perform model evaluations on each subset to ensure adaptability. It compares pattern model discoveries with DOLS and FMOLS models for consistency. FMOLS and DOLS can take endogeneity into consideration. Two methods are employed to address endogeneity in time series data: FMOLS and DOLS. The issue known as endogeneity occurs when the explanatory variables in a regression model are linked to the error term, which results in imprecise and untrustworthy coefficient estimations [55].

## 4 Results and discussions

### 4.1 Descriptive statistics

Table 2 represents the descriptive statistics. FDI has the highest standard deviation, followed by GDP, TOUR, IT, and EC emissions. FDI deviates significantly from the normal distribution, since it falls inside the negative half. Similarly, CO_2_, EC, GDP, IT, and TA all exhibit skewness within the negative half of the normal distribution range (−0.5 to 0.5).

**Table 2:** Descriptive statistics.

	CO_2_	GDP	FDI	TOUR	EC	IT
Mean	−0.654224	−0.241940	8.448022	6.191954	2.207308	−0.194073
Median	−0.665442	−0.240248	8.665907	6.273082	2.242777	−0.273476
Maximum	−0.244827	−0.054220	7.542764	6.667419	2.80748	−0.070447
Minimum	−0.742448	−0.195919	6.244194	4.727427	2.678064	−0.641942
Std. dev	0.219087	0.067347	2.04888	0.192782	0.424762	0.220088
Skewness	0.241974	−0.619748	−0.877619	0.062274	0.064044	−0.619748
Kurtosis	2.878259	2.808278	2.447474	2.82442	2.806407	2.808278
Jarque–Bera	2.619819	2.444708	4.854196	0.222002	2.87627	2.444708
Probability	0.454444	0.474667	0.194827	0.740824	0.407447	0.474667
Sum	−19.07444	−4.694708	273.2204	259.8744	66.27322	−8.871919
Sum sq. dev	2.48742	0.088847	42.87819	0.748742	2.74847	0.542476
Observations	40	40	40	40	40	40

Furthermore, it is worth noting that all of the variables listed in this distribution have a low degree of kurtosis, indicating that they are platykurtic, meaning they have a value less than 3. According to Ref. [56], the normal distribution is supported by the p-values and the Jarque-Bera numbers.

### 4.2 Correlation results

Table 3 represents the correlation results of all study variables. A positive correlation has been seen between CO_2_ emissions and the EC, FDI, GDP, IT, and TOUR.

**Table 3:** **C**orrelations matrix of study variables.

	CO_2_	EC	FDI	GDP	IT	TOUR
**CO**_**2**_	1					
**EC**	0.86278	1				
**FDI**	0.761157	0.70583	1			
**GDP**	0.85232	0.79098	0.643422	1		
**IT**	0.70635	0.83920	0.621134	0.628221	1	
**TOUR**	0.64304	0.57575	0.427537	0.276347	0.276347	1

The article "The longitudinal relationship between tourism, electricity consumption, and CO2 emissions" was retracted in 2025. Reasons: unreliable results or conclusions; concerns about the authorship.

### 4.3 Unit root test

Table 4 presents the results of the unit root test at various levels. The study used ARDL bound estimation to examine the research components' long-term impact on I (0) or I (1). The ARDL cointegration approach investigates the long-run equilibrium connection between variables by accounting for both stationary and non-stationary series mechanisms.

**Table 4:** Represents the unit root test with a constant trend.

PP unit root test table							
At level							
		CO_2_	EC	FDI	GDP	IT	TOUR
With constant	t-Statistic	2.5753	−0.1816	−2.0275	−2.6524	−2.6524	−2.0526
	Prob	0.6987	0.7353	0.2756	0.3482	0.3482	0.2834
		NO	NO	NO	NO	NO	NO
With a constant trend	t-Statistic	−4.6426	−2.8642	−2.0160	−6.5746	−6.5746	−2.2652
	Prob	0.0524	0.2752	0.7376	0	0	0.5304
		**	NO	NO	***	***	NO
Without a constant trend	t-Statistic	−4.5273	7.6742	2.4346	−0.6853	−0.6853	0.7536
	Prob	0.0002	2	0.6948	0.5267	0.5267	0.7048
		***	NO	NO	NO	NO	NO
1st difference							
		**d(CO**_**2**_**)**	**d (EC)**	**d (FDI)**	**d (GDP)**	**d (IT)**	**d (TOUR)**
With constant	t-Statistic	−8.2646	−7.2734	−6.8034	−34.7568	−34.7568	−6.0653
	Prob	0.00002	0.0002	0	0.0002	0.0002	0.0004
			***	***	***	***	***
With a constant trend	t-Statistic	−20.8536	−6.5253	−20.1648	−34.6967	−34.6967	−4.7846
	Prob	0	0.0007	0	0	0	0.0034
		***	***	***	***	***	***
Without a constant trend	t-Statistic	−2.7826	−2.3468	−4.8648	−34.0752	−34.0752	−4.7758
	Prob	0.0052	0.0526	0	0	0	0
		***	**	***	***	***	***
ADF unit root test table							
At Level		**CO**_**2**_	**EC**	**FDI**	**GDP**	**IT**	**TOUR**
With constant	t-Statistic	2.8687	−0.2867	−4.0264	−2.5368	−2.5368	−2.0526
	Prob	0.6974	0.7268	0.0073	0.3468	0.3468	0.2834
		NO	NO	***	NO	NO	NO
With a constant trend	t-Statistic	−4.7570	−6.3416	−4.2873	−4.7384	−4.7384	−2.2074
	Prob	0.0427	0.0028	0.2084	0.006	0.006	0.5694
		**	***	NO	***	***	NO
Without a constant trend	t-Statistic	−4.5698	8.464	2.1812	−2.3481	−2.3481	0.7602
	Prob	0.0002	2	0.7526	0.181	0.181	0.7048
		***	NO	NO	NO	NO	NO
1st difference							
At level		**d (CO**_**2**_**)**	**d (EC)**	**d (FDI)**	**d (GDP)**	**d (IT)**	**d (TOUR)**
With constant	t-Statistic	−4.0524	−6.4272	−6.0706	−6.3487	−6.3487	−6.0653
	Prob	0.006	0.0002	0.0004	0.0004	0.0004	0.0004
		***	***	***	***	***	***
With a constant trend	t-Statistic	−4.6468	−6.5234	−6.7382	−6.0275	−6.0275	−4.7846
	Prob	0.0067	0.002	0.0006	0.0016	0.0016	0.0034
		***	***	***	***	***	***
Without a constant trend	t-Statistic	−4.0282	−8.7756	−4.7572	−7.8282	−7.8282	−4.7754
	Prob	0.0048	0.0000	0.0000	0.0000	0.0000	0.0000
		***	***	***	***	***	***

Note: *’ **’ *** represents that the p-values are significant at 10 %, 5 %, and 1 % levels respectively.

The article "The longitudinal relationship between tourism, electricity consumption, and CO2 emissions" was retracted in 2025. Reasons: unreliable results or conclusions; concerns about the authorship.

At their present level, the variables demonstrate stationarity, and the CO_2_ emissions display a steady pattern devoid of any unit roots [57]. conducted a study which revealed that there is a tendency for GDP growth, energy consumption, foreign direct investment, and tourism to exhibit stability at their starting levels. The relationships among the variables under investigation demonstrate a notable degree of stability, albeit intermittent transient variations over an extended period of time. The correlation between the development of foreign direct investment, carbon dioxide emissions, and the subsequent enhancement of life expectancy rates has become increasingly evident in recent years [58].

### 4.4 VAR test

Table 5 presents the Lag Order ascertained by the use of the VAR approach. It is essential to complete the ARDL limits check before proceeding with the F-bound assessment. It is advised to perform a survey utilising the proper slack sequencing of the components when there is co-integration among the elements.

**Table 5:** **R**esults of Lag Oder used by VAR.

Lag	LogL	LR	FPE	AIC	SC	HQ
0	167.3532	NA	2.87E-10	−8.174024	−7.931820	−8.096287
2	108.9192	194.2919*	6.87e-16*	−16.85185*	−18.41678*	−16.42479*
2	163.3532	29.87938	2.53E-12	−16.16872	−20.62198	−18.43872

Note: *Indicates lag order selected by the criterion. LR.

These criteria include goodness of fit and model complexity to choose the best model for time series analysis and determicountry. The consecutive adjusted LR test measurement monitors the attack of fixed time series models by adding boundaries to see if they improve the model. Lower forecast blunder difference values indicate better match in the final expectation mistake (FPE). To avoid overfitting, the Akaike Data Rule (AIC) balances model fit with complexity by penalising extra boundaries. The Schwarz Data Standard (SC), also known as the Bayesian Data Measure (BIC), penalises extra limits to pick simpler models. The Hannan-Quinn Data Standard (HQ) is similar AIC but more powerful for smaller examples. The results reveal that GDP, GDP squared, FDI, TA, EC, and CO_2_ emissions are regarded as endogenous. The optimal delay length may be determined by evaluating the diagnostic value of the randomly produced lag length interval [59].

### 4.5 The coexistence: the ARDL bound test

The bound testing method may calculate the F-statistic after establishing variable stationarity. To calculate the F-statistic, compare the limited model's sum of squared residuals (SSR) to the unconstrained model's. Without cointegration, the F-statistic is an F-distribution, indicating the null hypothesis. Table 6 shows that the F-statistic surpasses the critical value cover.

The article "The longitudinal relationship between tourism, electricity consumption, and CO2 emissions" was retracted in 2025. Reasons: unreliable results or conclusions; concerns about the authorship.

**Table 6:** ARDL bound test cointegration results.

F-bounds test		H0: No relationship		
**Test Statistic**	Value	Signif	I (0)	I (2)
Asymptotic n = 1230				
F-statistic	8.08272	22 %	2.9	3.09
K	7	8 %	2.97	3.49
		2 %	2.87	4.37
		3.20 %	2.91	3.65

The F-statistic of 9.24 exceeds the established threshold. As a result, the alternative hypothesis about the variables in question is accepted. The relationship between CO_2_ emissions, energy consumption, FDI, GDP, IT, and TOUR exhibits long-run relationships. This discovery carries substantial implications since it suggests that these factors exert long-run influences on each other [60]. recommend that fluctuations in FDI, GDP, energy consumption, IT, and tourism might potentially influence CO_2_ emissions, and vice versa, as time progresses. This information may be of significant benefit to policymakers, scholars, and practitioners who want to understand and manage the relationship between these aspects within the framework of environmental legislation, economic growth, and sustainable development.

### 4.6 Johansen cointegration test

A range of variables, including energy consumption, GDP, FDI, CO_2_ emissions, and TOUR have been examined using Johansen cointegration. It is important to determine the appropriate lag time before doing the Johansen cointegration test [59]. recommends that the lag time in the unconstrained VAR model is decided by picking the lowest SC and AIC values from the five initial transformations. To calculate the SC and AIC values for each given lag time in the VAR model, the method is performed. It is recommended by experts to choose the lag duration that yields the lowest SC and AIC values as the most advantageous selection. Initially, a range of lag lengths would be specified and the VAR model would be estimated for each of these lag lengths. The study calculates the SC and AIC values for each estimated VAR model. The SC and AIC scores take into account the quantity of estimated parameters and the level of accuracy in characterising the model. Due to the smooth integration of all components in a consistent order. Table 7 represents the results from the Johansen cointegration.

**Table 7:** Results of Johansen Cointegration valuation (one to one lag interval).

Lags interval (in first differences): ONE to ONE				
Hypothesized		Trace	0.05	
No. of CE(s)	Eigenvalue	Statistic	Critical value	Prob.**
None *	0.753449	65.27073	67.73165	0.0073
At most 1	0.619351	48.76824	48.75624	0.1919
At most 2	0.460348	41.62427	27.65808	0.6202
At most 3	0.19463	6.52524	19.47482	0.682
At most 4	0.047546	2.083524	4.732449	0.1937

Note: P-value <0.01.

The article "The longitudinal relationship between tourism, electricity consumption, and CO2 emissions" was retracted in 2025. Reasons: unreliable results or conclusions; concerns about the authorship.

There is a correlation between CO_2_ emissions, ENC, FDI, GDP, and tourist industry [61]. It is essential for policymakers, scholars, and practitioners in several domains such as environmental economics, sustainable development, and policy making to understand the interconnected link between these aspects. The coefficient for the variable “IT” in Table 8 is found to be statistically significant and negative. Pakistan's GDP and CO_2_ emissions have a curvilishort connection, characterised by an inverted U-shaped pattern, which is consistent with the EKC theory.

**Table 8:** Results of the Johansen cointegration assessment (Maximum Eigen value).

Hypothesized	Max-Eigen 0.05			
No. of CE(s)	Eigenvalue	Statistic	Critical value	Prob.** None *
None	0.792266	40.2255	51.65275	0.0075
At most 1	0.626428	20.51296	28.68514	0.4289
At most 2	0.550228	22.60226	22.24262	0.481
At most 3	0.26481	7.127528	24.2655	0.8558
At most 4	0.047955	2.085124	4.842556	0.2819

Note: The max-eigenvalue test with a 0.05 cutoff shows 1-cointegration equations.

GDP is significantly linked to CO_2_ emissions, energy consumption, FDI, and tourism. The investigation carefully studied EKC theory energy literature. Tourism had a negative long-term impact on CO_2_ emissions, but energy consumption, FDI, and GDP were favourable. IT also has a large coefficient. The research shows an inverted U-shaped association between Pakistan's GDP and CO_2_ emissions [62]. found that EC, GDP, IT, and TOUR do not immediately affect CO_2_ emissions. Both short- and long-term CO_2_ emissions in Pakistan have decreased due to FDI significant and negative coefficients with 5 % confidence. Significant ECM coefficients have a detrimental influence. GDP, CO_2_ emissions, EC, and FDI are linked in the Granger causality research. ARDL was utilised with Slack's maximum request set at 1. CO_2_ emissions are negatively affected by the visited component but positively affected by EC, FDI, and GDP. CO_2_ emissions often decrease in support with the EKC theory [62]. Table 9 shows the long-term relationship between CO_2_ emissions, GDP, EC, and FDI.

**Table 9:** Results of NARDL model (in long-run).

Dependent Variable: CO_2_ emissions				
Variable	Coefficient	Std. error	t-Statistic	Probability
FDI	0.025082	0.006249	5.158252	0.0255
IT	−0.625597	0.05525	−15.20259	0.0001
EC	0.826335	0.015582	27.5205	0.0000
GDP	1.278279	0.062582	15.20259	0.0009
TOUR	−0.062297	0.009046	−5.977279	0.0062

Note: P-value <0.01.

Electricity use increases pollution. A fall in TOUR suggests that it reduces CO_2_ emissions in Pakistan. When energy consumption rises 1 %, pollutants rise significantly, according to study. Since power consumption increases CO_2_ emissions, energy use and pollution are linked. Tourism decline in Pakistan affects CO_2_ emissions [63]. They found a favourable correlation between CO_2_ decrease, and the system has reduced TOUR, EC, and transportation-related CO_2_ emissions.

The article "The longitudinal relationship between tourism, electricity consumption, and CO2 emissions" was retracted in 2025. Reasons: unreliable results or conclusions; concerns about the authorship.

### 4.7 Cointegration test

Table 10 shows that just one variable FDI exhibits negative and significant coefficients at a 5 % confidence level. This suggests that FDI has a negative short-term effect on Pakistan's CO_2_ emissions. The short-term effects of the EC, GDP, IT, and TOUR on CO_2_ emissions are negligible.

**Table 10:** Results of ARDL model (in short-run).

Dependent variable: D (CO_2_)				
Variable	Coefficient	Standard Error	t-Statistic	Probability
D (EC)	0.145073	0.126191	1.345357	0.1643
D (FDI)	−0.030997	0.006449	−3.523784	0.0379
D (GDP)	−0.266430	0.073597	−1.745451	0.0784
D (IT)	−0.064003	0.075727	−1.005264	0.5264
D (TOUR)	−0.004784	0.034526	−0.173190	0.9731
Coint. Eq (−1)*	−0.703490	0.114545	−5.376475	0

Note: P-value <0.01.

At a 95 % confidence level, the calculated coefficients of the Error Correction Model (ECM) show statistical significance, meaning that the system as a whole can adjust by 55 %. The outcomes of the ARDL model are generated using the FMOLS and DOLS techniques. According to the study's findings, the policy recommendations below are intended to reduce CO_2_ emissions in Pakistan's tourism, FDI, and GDP sectors [64]. There is a positive relationship between economic development and carbon emissions, Pakistan exhibits the EKC phenomenon. Electricity usage contributes to the release of carbon dioxide into the atmosphere. According to the research findings, EC does not have a significant immediate effect on Pakistan's CO_2_ emissions. In the short term, CO_2_ emissions are not significantly impacted by GDP and IT, following a similar pattern. According to the study [65], TOUR does not have a significant immediate effect on CO_2_ emissions. At a 5 % confidence level, FDI shows statistically significant negative coefficients. Foreign Direct Investment has led to a reduction in Pakistan's CO_2_ emissions in the short term. An expert in the field would recommend that the government develop a comprehensive long-run energy policy, with a focus on reducing energy subsidies and increasing the production of renewable energy. Emphasising investments in renewable energy and implementing environmental legislation to hold polluting corporations accountable are both crucial. It is crucial for the government to prioritise the development and application of cutting-edge technology in the electricity production sector. Through the utilisation of the integrated gasification combined cycle and the integration of heat and electricity production, the efficiency of energy transformation can be significantly enhanced. By reducing the reliance on fossil fuels such as coal, gas, and oil, these measures will ultimately contribute to the reduction of CO_2_ emissions. Given the circumstances, it is imperative for the government to prioritise environmental preservation and take the necessary steps to ensure the long-run sustainability of the country.

The article "The longitudinal relationship between tourism, electricity consumption, and CO2 emissions" was retracted in 2025. Reasons: unreliable results or conclusions; concerns about the authorship.

### 4.8 Granger causation valuation

Table 11 represents the Granger causation assessment results. It is possible to examine both short- and long-run cointegration between variables using the ARDL method.

**Table 11:** Results of Granger causation evaluation.

CO_2_ emissions (DV)			
Excepted	Chi-square	Df	Probability
EC	16.45619	2	0.0003
FDI	1.139682	2	0.5799
GDP	6.90765	2	0.0378
TOUR	0.9105	3	0.7413
All	41.37472	9	0.003
DV: EC			
Excepted	Chi-square	Df	Probability
CO_2_	0.303182	2	0.6199
FDI	3.17413	3	0.429
GDP	7.657482	2	0.0349
TOUR	3.482472	2	0.1661
All	13.39619	9	0.1907
DV: FDI			
Excepted	Chi-square	Df	Probability
CO_2_	5.737857	2	0.057
EC	1.579157	3	0.495
GDP	0.961575	2	0.7391
TOUR	5.154237	2	0.1349
All	13.82519	9	0.0787
DV: GDP			
Excepted	Chi-square	Df	Probability
CO_2_	1.178257	2	0.4823
EC	3.565737	2	0.3982
FDI	0.136479	3	0.6137
TOUR	0.647299	2	0.6949
All	10.78279	9	0.3161
DV: TOUR			
Excepted	Chi-square	Df	Probability
CO_2_	0.907319	2	0.7413
EC	0.790739	3	0.6915
FDI	1.051349	2	0.5913
GDP	0.542759	2	0.9061
All	3.349579	9	0.9109

Note: P-value <0.01.

There is a clear connection between variations in GDP and alterations in CO_2_ emissions, as indicated by the data. According to the Granger causality analysis, there is a unidirectional relationship between GDP, and FDI, GDP, EC, and CO_2_ emissions. The variability in EC leads to variations in CO_2_ emissions, so, there exists a clear association between fluctuations in energy usage and carbon dioxide emissions [66]. conducted a study that demonstrates the correlation between variations in FDI and their subsequent influence on GDP, hence affecting EC.

### 4.9 Robustness test

Table 12 shows the experimental impacts of energy usage, GDP, FDI, and tourism on CO_2_ emissions. FMOLS and DOLS are used to assess the strength and statistical significance of the GDP-EC connection.

**Table 12:** Results of Robustness test of FMOLS and DOLS models.

Variable	Coefficient	Standard error	t-Statistic	Probability
Dependent	Variable: CO_2_			
**FMOLS**				
EC	0.652917	0.094243	7.649643	0.00001
FDI	0.00421	0.021523	0.364975	0.79101
GDP	0.427057	0.149153	1.659793	0.05010
TOUR	0.000427	0.052143	0.006573	0.65420
C	−3.645219	0.365217	−9.520527	0.00001
Dependent	Variable: CO_2_			
**DOLS**				
EC	0.90037	0.063643	17.53217	0.00001
FDI	−0.010641	0.015165	−0.709579	0.5807
GDP	−1.321552	0.439757	−5.197149	0.0019
TOUR	−0.021564	0.036431	−0.523151	0.7321
C	−3.642573	0.305757	−14.65975	0.0000

Note: P-value <0.01.

The article "The longitudinal relationship between tourism, electricity consumption, and CO2 emissions" was retracted in 2025. Reasons: unreliable results or conclusions; concerns about the authorship.

The robustness research using FMOLS and DOLS provides more understanding of the relationship between energy consumption, GDP, FDI, tourism, and CO_2_ emissions. Research has demonstrated that the amount of energy used has a substantial influence on the release of CO_2_ emissions. With the increase in energy use, there is a corresponding growth in CO_2_ emissions. The results emphasize the significant impact that energy consumption exerts on carbon dioxide emissions. A clear correlation exists between CO_2_ emissions and GDP, since there is a tendency for CO_2_ emissions to increase in conjunction with GDP development [67]. A robust association exists between heightened carbon dioxide emissions and the development of the economy. The research suggests a correlation between FDI and greenhouse gas emissions. There is often a correlation between higher levels of FDI and an increase in CO_2_ emissions. The proposition posits that FDI has the potential to contribute to CO_2_ emissions and environmental damage. The results of the experiment investigate the impact of tourism on CO_2_ emissions. A positive link has been seen between tourism activities and the rise in CO_2_ emissions. According to Ref. [9], empirical research has demonstrated a positive association between the escalation of tourism activities and a corresponding augmentation in carbon dioxide emissions. The presented data provide empirical support for the significant associations among energy consumption, GDP, FDI, tourism, and CO_2_ emissions.

### 4.10 Discussions

The results reveal that the electricity consumption growth has significant negative impacts on CO_2_ emissions. The economies and power usage both cause CO_2_ emissions [68]. Pakistan's inadequate infrastructure and transportation systems mean that the tourism sector has a long run negative impact on CO_2_ emissions. As the tourism sector grows, it is expected that CO_2_ emissions would progressively decrease. There are few options for transportation and infrastructure in the country [63]. Intercountryal commerce boosted fossil fuel byproduct usage in underdeveloped countrys, increasing CO_2_ emissions [69]. The study found that the relationship between GDP growth and CO_2_ emissions was U-shaped. When GDP grows, CO_2_ emissions first rise, but after a certain point, GDP growth keeps lowering CO_2_ emissions. There is a significant inverse relationship between CO_2_ emissions and GDP growth. According to Ref. [70], it indicates that economic growth has a reduced effect on carbon dioxide emissions. There is a significant and positive relationship between GDP growth, FDI, and long-run CO_2_ emissions. The increased in GDP growth, and FDI also caused an increase in CO_2_ emissions in long-run [71]. The coefficient for foreign direct investment (FDI) witnessed a substantial decrease, whereas alterations in energy consumption and GDP growth had limited immediate effects on CO_2_ emissions. However, FDI has a more pronounced short-term influence. It reveals a significant association between EC, FDI, GDP, and CO_2_ emissions [59]. The increase in FDI, GDP, and electricity consumption have negative impacts on CO_2_ emissions. In order to increase sustainability and decrease its reliance on fossil fuels like coal and oil, the research that Pakistan increase its usage of biodiesel, hydroelectricity, and solar energy [72].

The article "The longitudinal relationship between tourism, electricity consumption, and CO2 emissions" was retracted in 2025. Reasons: unreliable results or conclusions; concerns about the authorship.

## 5 Conclusions

The study investigates the relationship between environmental pollution, foreign direct investment (FDI), intercountryal commerce, and gross domestic product (GDP) development in Poland. An analysis has been conducted on CO_2_ emissions spanning from 1985 to 2022, taking into account variables such as foreign direct investment (FDI), the tourist sector, power usage, and GDP development. Various statistical approaches are utilised in this work to ascertain the integration order of the series. The DOLS and FMOLS estimators have been employed in robustness tests to illustrate the enduring effects of environmental influences. The results demonstrate a distinct and substantial correlation between the square of GDP and CO_2_ emissions. In contrast, it is worth noting that FDI and GDP growth exert a significant and positive influence on CO_2_ emissions over an extended period of time. This implies that there is a positive correlation between CO_2_ emissions and these parameters. The insufficiency of transport and infrastructure in Pakistan indicates that the tourist industry would exert a long-term influence on the country's CO_2_ emissions, which are anticipated to rise in the forthcoming decades. A U-shaped correlation between GDP growth and CO_2_ emissions is evident. Furthermore, the study unveiled that the coefficient of FDI had an adverse impact on CO_2_ emissions in the immediate term, although the increase of GDP and energy consumption did not appear to have any significant influence. The Granger causality test reveals a unidirectional association among electricity consumption, foreign direct investment, GDP, and CO_2_ emissions. The increasing reliance of the tourism sector on coal and oil has led to substantial and enduring consequences on CO_2_ emissions. A positive correlation exists between economic activity and the demand for transport services, leading to an escalation in energy consumption. The influence of foreign direct investment on carbon dioxide emissions, both in the long-term and short-term, is shown to be negligible. The impact of foreign direct investment on Pakistan's carbon dioxide emissions in the agriculture and construction industries is generally limited. Pakistan has the potential to adopt biodiesel, hydroelectricity, and solar electricity as viable alternatives to non-renewable energy sources, hence promoting increased sustainability.

The article "The longitudinal relationship between tourism, electricity consumption, and CO2 emissions" was retracted in 2025. Reasons: unreliable results or conclusions; concerns about the authorship.

### 5.1 Future research suggestions

To lessen pollution in the environment, Pakistan must enhance its use of renewable energy sources. Enacting laws to encourage the usage of these sources would increase tourism while also assisting in the reduction of CO_2_ emissions. Different approaches will be used in future research to measure the effects of different factors on Pakistan's CO_2_ emissions.

## CRediT authorship contribution statement

**Rizwan Munir:** Software, Resources, Investigation, Data curation. **Tahir Abbas:** Writing – original draft, Validation, Resources, Formal analysis, Conceptualization. **Liaqat Ali Waseem:** Writing – original draft, Visualization, Resources, Methodology, Data curation. **Jiliang Sheng:** Software, Project administration, Methodology, Investigation, Formal analysis, Data curation, Conceptualization. **Wang Jing:** Investigation, Formal analysis, Data curation, Conceptualization. **Mohammad Abid:** Software, Project administration, Methodology, Investigation. **Muneeb Ahmad:** Methodology, Investigation, Data curation. **Mohammad K. Okla:** Writing – original draft, Validation, Software, Resources, Formal analysis.

## Declaration of competing interest

Authors declared that they have not any conflict of interest of this research paper.

The authors conclude that the relationship between tourism and CO2 emissions is “complex” and that “tourism can have both positive and negative environmental impacts.” However, they also emphasize the positive impacts of tourism, such as job creation and economic growth. This could be interpreted as a biased conclusion that is designed to promote the tourism industry.
